# *Cistanche deserticola* polysaccharides alleviate cognitive decline in aging model mice by restoring the gut microbiota-brain axis

**DOI:** 10.18632/aging.203090

**Published:** 2021-06-03

**Authors:** Yuan Gao, Bing Li, Hong Liu, Yajuan Tian, Chao Gu, Xiaoli Du, Ren Bu, Jie Gao, Yang Liu, Gang Li

**Affiliations:** 1 Inner Mongolia Medical University, Hohhot 010110, China; 2 Shanxi Key Laboratory of Chinese Medicine Encephalopathy, Shanxi University of Chinese Medicine, Jinzhong 030619, China

**Keywords:** learning and memory deterioration, CDPS, gut microbiota

## Abstract

Recent evidence suggests alterations in the gut microbiota-brain axis may drive cognitive impairment with aging. In the present study, we observed that prolonged administration of D-galactose to mice induced cognitive decline, gut microbial dysbiosis, peripheral inflammation, and oxidative stress. In this model of age-related cognitive decline, *Cistanche deserticola* polysaccharides (CDPS) improved cognitive function in D-galactose-treated mice by restoring gut microbial homeostasis, thereby reducing oxidative stress and peripheral inflammation. The beneficial effects of CDPS in these aging model mice were abolished through ablation of gut microbiota with antibiotics or immunosuppression with cyclophosphamide. Serum metabolomic profiling showed that levels of creatinine, valine, L-methionine, o-Toluidine, N-ethylaniline, uric acid and proline were all altered in the aging model mice, but were restored by CDPS. These findings demonstrated that CDPS improves cognitive function in a D-galactose-induced aging model in mice by restoring homeostasis of the gut microbiota-brain axis, which alleviated an amino acid imbalance, peripheral inflammation, and oxidative stress. CDPS thus shows therapeutic potential for patients with memory and learning disorders, especially those related to gut microbial dysbiosis.

## INTRODUCTION

Prolonged administration of D-galactose (D-gal) and beryllium salts induces aging in experimental animal models and *in vitro* primary cell cultures and is used to identify mechanisms underlying the natural aging process [1–4]. Previous studies show that cognitive decline in D-galactose-induced aging model mice is related to reduced nerve growth factor (NGF) protein levels and increased reactive oxygen species (ROS) in the brain, both of which cause degeneration of the hippocampal neurons and reduce neurogenesis [3, 4]. Recent studies have also shown that the composition and number of human gut microbiota significantly changes during the aging process [5].

*Cistanche deserticola* is an herb that grows mainly in the North-Western desert region of China and is used in traditional Chinese medicine. It is commonly known as “ginseng of the desert.” *Cistanche deserticola* extracts contain several pharmacologically active compounds, including phenylethanoid glycosides, iridoids, lignose, oligosaccharides, polysaccharides, and amino acids; these compounds are associated with anti-inflammatory, anti-oxidative, anti-senescent, neuroprotective, and immunomodulatory properties [6, 7]. For example, polysaccharides extracted from *Cistanche deserticola* have been used in traditional Chinese medicine to treat colorectal cancer [8]. A wide range of weakly toxic polysaccharides with useful bioactivities have been isolated from several organisms, such as Chuanqiong polysaccharide, Ganoderma lucidum polysaccharide, and Lycium barbarum polysaccharide [9–11]. CDA-0.05 is a galactoglucan isolated from *Cistanche deserticola* that promotes growth of several beneficial intestinal bacteria, including several species of *Bacteroides* and *Lactobacillus* [12].

The underlying mechanisms of the normal aging process are also implicated in several human diseases such as neurodegenerative disorders, coronary atherosclerosis, type 2 diabetes (T2DM), and hypertension [13, 14]. Recent studies have shown that changes in the intestinal flora play a significant role in human aging [15]. Several studies have shown that prolonged administration of D-galactose in experimental mice and rats mimics normal aging process and is a useful model to study aging-related phenotypes such as cognition decline [16]. Moreover, D-galactose-induced aging model mice show changes in the composition of gut microbiota [17]. Therefore, we hypothesized that changes in the gut microbiota composition may cause cognitive decline in the D-galactose-induced aging model mice, and investigated if *Cistanche deserticola* polysaccharides (CDPS) may alleviate cognitive decline by restoring gut microbiota dysbiosis.

## RESULTS

### D-galactose-induced aging model mice demonstrate cognitive decline and gut microbial dysbiosis

We analyzed behavioral performance of wild-type (WT) mice and those treated with 150 mg D-gal per Kg body weight for 2 months (model or Mod) using novel object recognition and Morris water maze (MWM) tests. The preferential index values in the novel object recognition test were significantly reduced in the Mod group mice compared to the WT group mice (Figure 1A, 1B). MWM test results showed that the escape latency time after sixth day was significantly increased in the Mod group compared to the WT group (Figure 1C, 1D). Moreover, target platform crossings and swimming times within the target quadrant were significantly reduced in the Mod group compared to the WT group (Figure 1E, 1F). These results demonstrated significant decline in the learning and memory abilities of the D-gal-induced aging model mice.

**Figure 1:** **Prolonged administration of D-galactose induces learning and memory impairment in mice.** (**A**, **B**) Novel object recognition test results show preferential index values for WT and model group mice after (**A**) 24 h training and (**B**) 1 h testing phase. (**C**–**F**) Morris water maze test results show (**C**) latency in learning phase, (**D**) latency in test phase, (**E**) number of plate crossings, and (**F**) time in the target quadrant for the WT and model group mice. Note: *p<0.05, **p<0.01, ***p<0.001 compared with the WT group mice; by. All values are represented as means ± SEM (n=15); Data was analyzed by one-way ANOVA followed by Dunnett's post hoc test.

We then analyzed the differences in the abundance and composition of the gut microbial phyla, genera and species in the fecal samples of the Mod and WT groups of mice using 16S ribosomal RNA (rRNA) sequencing data from fecal samples. The predominant intestinal flora in the WT and Mod group mice were *Firmicutes* and *Bacteroides*. However, the abundance of *Bacteroides* was significantly reduced and the abundance of *Firmicutes* was significantly increased in the Mod group compared to the WT group (Figure 2A). Next, we performed linear discriminant analysis (LDA) to determine LDA effect size (LEfSe) scores followed by Kruskal-Wallis and Wilcoxon tests to evaluate the relative abundance of different taxa in the WT and Mod group mice. The LDA results are shown in Figure 2B. Furthermore, we constructed cladograms showing differential enrichment of various genera and species belonging to the Bacteriodes and Firmicutes phyla in the WT and model groups (Figure 2C). Overall, our results demonstrated impaired cognitive ability and gut microbial dysbiosis in the D-galactose-induced aging model mice.

**Figure 2:** **Prolonged administration of D-galactose induces gut microbial dysbiosis in mice.** (**A**) The relative abundance of the top 10 gut microbial phyla in the WT and Mod group mice. (**B**) The relative abundance of the gut microbial genera based on the linear discriminant analysis (LDA) scores in the WT and Mod group mice. (**C**) LEfSe cladogram shows the most enriched gut bacterial genera in the WT and Mod group mice. Only taxons with LDA scores >4 and p-value <0.05 are represented in (**B**, **C**). Note: All data are represented as means ± SEM (n=15). The differences between groups were analyzed by unpaired Student's t-tests.

### CDPS treatment improves cognitive ability in the D-gal-induced aging model mice

We analyzed if CDPS treatment alleviates cognitive decline in D-gal-induced aging model mice. During the 2 months of administration, the body weight was measured every other day. The body weights of the model and CDPS groups of mice were similar (Figure 3A). Conduct behavioral experiments after the last dose. Novel object recognition and Morris water maze test results showed that short-term memory was significantly higher in the CDPS groups of mice compared to the model group of mice; long-term memory in the CDPS group of mice was higher but statistically insignificant compared to the model group of mice (Figure 3B, 3C). This suggested that CDPS treatment abrogated loss of short-term object recognition memory in D-gal treated mice.

**Figure 3:** **CDPS treatment improves learning and memory in the D-gal aging model mice.** (**A**) The body weights of WT, Mod, and CDPS group mice during administration. (**B**, **C**) Novel object recognition test results show the preferential index in WT, Mod, and CDPS group mice after (**B**) 24 h training and (**C**) 1 h testing phase. Morris water maze test results show (**D**, **E**) escape latency, (**F**) number of plate crossings, and (**G**) time in the target quadrant for the WT, Mod, and CDPS group mice. Note: *p<0.05, **p<0.01, and ***p<0.001 compared to the WT group mice; #p<0.05, ##p<0.01, and ###p<0.001 compared to the Mod group mice. Differences between groups were analyzed by one-way ANOVA followed by the Dunnett's post hoc test. All values are shown as means ± SEM (n=15).

The spatial learning and memory of these mice were evaluated by Morris water maze test, and the results showed that the escape latency times of the CDPS group of mice were comparable to the WT group of mice and significantly shorter than the Mod group mice (Figure 3D). Furthermore, escape latency times were significantly lower on the sixth day post-CDPS administration compared to the model group (Figure 3E). The swimming time within the target quadrant was significantly higher in the CH and CM groups compared to the model group. The CL group is higher than the model group but no statistical significance (Figure 3F). Moreover, the number of platform crossings was significantly higher in the CM and CL groups compared to the model group. However, the CH group is higher than the model group and no statistical significance (Figure 3G). These results demonstrated that CDPS treatment improved spatial learning and memory in the D-gal-induced aging model mice.

### CDPS treatment restores homeostasis of the gut microbiota composition in the D-galactose-aging model mice

Monosaccharides and polysaccharides are the essential nutrients required for the growth of bacteria [18–21]. It is also reported that CDPS regulates the composition of gut microbiota [22]. Therefore, we analyzed if CDPS treatments alleviated the gut microbial dysbiosis in the model group mice by evaluating16S rRNA sequencing data of feces samples from the WT, model, and CDPS groups of mice.

First, we calculated alpha diversity indices to evaluate the overall fecal microbiota richness and structural difference among these groups. We analyzed alpha diversity (α-diversity) indexes such as observed species, Shannon, Chao 1, ACE, and Simpson index values to determine changes in the composition of various bacterial species in the feces samples of different murine groups. The α-diversity (observed species, Shannon, Chao 1, ACE and Simpson indexes) indexes were higher in the WT and CDPS groups of mice compared to the model group, but statistical significance was only observed for the Chao 1 index values between the CM group and Mod group. It indicated that administration with CDPS increases the microbiome richness (Figure 4A–4E). Next, we analyzed β-diversity indexes to identify differences in the gut microbial species between the WT, model, and CDPS groups of mice using Non-metric Multidimensional Scaling (NMDS), Principal Coordinates Analysis (PCoA), and Principal Component Analysis (PCA). PCA showed variations in the gut microbial composition of the model group mice during the aging process, including dimension reduction and maintenance of patterns and trends (Figure 4F). The differences in the fecal microbiota between the WT, model, and CDPS groups were identified based on PCoA of the unweighted UniFrac distances for the 16S rRNA genes (Figure 4G). Clustering analysis showed significant differences in NMDS between the model group and the WT and CDPS groups (Figure 4H).

**Figure 4:** **CDPS treatment restores gut microbial composition in the D-galactose-induced aging model mice.** (**A**–**E**) The α diversity indexes of the gut flora in the feces of WT, Mod, and CDPS (CH, CM, and CL) group mice. (**F**–**H**) The β diversity indexes show differences in the gut microbial species between WT, Mod, CH, CM, and CL groups of mice. (**I**) The relative abundance of top10 gut bacterial phyla in the WT, Mod, CH, CM, and CL groups of mice. (**J**) The top 100 gut microbial genus in the WT, Mod, CH, CM, and CL groups of mice. (**K**) The heatmap shows differentially enriched gut microbiota in the WT, Mod, CH, CM, and CL groups of mice. Note: *p<0.05, **p<0.01, and ***p<0.001 compared to the WT group mice; #p<0.05, ##p<0.01, and ###p<0.001 compared to the Mod group mice; Data were analyzed by unpaired Student's t-tests. All values are shown as means ± SD (n=15).

We evaluated the top 10 phyla of the gut microbiota and found that the abundance of the Bacteroides phyla was significantly higher in the CH, CM and CL group compared to the model group (Figure 4I). This suggested that CDPS restored the homeostasis of the gut microbiota in D-gal-treated mice. The cladograms showed differential enrichment of various genera and species belonging to *Bacteriodes* and *Firmicutes* phyla in the WT, model, and the CDPS groups (Figure 4J). As shown in the heatmaps, CDPS treatments reduced the relative abundances of *Thermoplasmata, Bacilli*, *unidentified Actinobacteria*, *Fusobacteriia* and *unidentified Elusimicrobia* and increased the relative abundances of *Methanobacteria, Spirochaetia, Deltaproteobacteria, unidentified_Deferribacteres, Mollicutes, Nitrososphaeria, Anaerolineae, Erysipelotrichia* and *unidentified_Cyanobacteria* compared to the model group (Figure 4K). These results demonstrated that CDPS treatment significantly restored homeostasis of the gut microbiota in the D-gal-induced aging model mice.

### CDPS treatment alleviates neurodegeneration in the D-gal-induced aging model mice by reducing oxidative stress

We next analyzed the effects of CDPS on inflammation by analyzing the serum levels of pro-inflammatory cytokines (IL-2 and TNF-α), and anti-inflammatory cytokines (IL-4 and IL-10) in different groups of mice. The serum levels of IL-2 and TNF-α were significantly lower and the serum levels of IL-4 and IL-10 were significantly higher in the CH, CM and CL group compared to the model group. It shown that CDPS has anti-inflammatory effects (Figure 5A–5D).

**Figure 5:** **CDPS treatment modulates circulating levels of pro- and anti-inflammatory cytokines and oxidative stress-related factors in the D-galactose-induced aging model mice.** ELISA assay results show serum levels of (**A**) TNF-α, (**B**) IL-2, (**C**) IL-4, (**D**) IL-10, (**E**) SOD and (**F**) MDA in the WT, Mod, and CDPS (CH, CM, and CL) group mice. Note: *p<0.05, **p<0.01, and ***p<0.001 compared to the WT group mice; #p<0.05, ##p<0.01, and ###p<0.001 compared to the Mod group mice. The data were analyzed by one-way ANOVA followed by Dunnett's post hoc test. All values are shown as means ± SEM (n=15).

Oxidative stress is caused by increased production of reactive oxygen species (ROS) and is one of the main factors that promotes aging [23]. Therefore, we analyzed the effects of CDPS on oxidative stress in the D-gal-induced aging mouse model by evaluating serum levels of the antioxidant enzyme, SOD, and the lipid peroxidation product, malondialdehyde (MDA). The serum levels of MDA were significantly higher and the serum levels of SOD were significantly reduced in the Mod group compared to the WT group, but, CDPS treatment reversed these effects (Figure 5E, 5F). These results demonstrated that oxidative stress was elevated in the D-gal-induced aging model mice, but was reduced by CDPS treatment.

Furthermore, we assessed the oxidative stress levels in the brain tissues by analyzing the levels of advanced oxidized protein product (AOPP), direct lipid peroxidation (LPO), and MDA as well as activities of antioxidant enzymes such as glutathione peroxidase (GSH-Px) and superoxide dismutase (SOD) in the brain tissue homogenates. The brains of Mod group mice showed significantly reduced activities of SOD and GSH-PX and significantly increased levels of AOPP, LPO and MDA compared to the WT group, but these effects were reversed in the CH, CM and CL group (Figure 6A–6E).

**Figure 6:** **CDPS treatment reduces oxidative stress in the brains of D-galactose-induced aging model mice.** (**A**–**E**) Colorimetric assay results show (**A**) AOPP, (**C**) LOP, and (**E**) MDA levels as well as (**B**) GSH-Px and (**D**) SOD enzyme activities in the brain homogenates of WT, Mod, and CDPS (CH, CM, and CL) group of mice. (**F**) Representative images (top to bottom: 40×, 100×, 400×; scale bar=100μm) show H&E and Nissl stained brain sections of WT, Mod, and CDPS (CH, CM, and CL) group mice. Note: *p<0.05, **p<0.01, and ***p<0.001 compared to the WT group mice; #p<0.05, ##p<0.01, and ###p<0.001 compared to the Mod group mice. The data were analyzed by one-way ANOVA followed by Dunnett's post hoc test. All values are shown as means ± SEM (n=15).

Furthermore, we performed histological staining of brain section with H&E and Nissl stains to assess the protective effects of CDPS on the brains of D-gal-induced aging model mice. The Mod group mice showed significant reduction in the neuronal numbers and volume, increased gap between neurons, irregular arrangement of neurons, and nuclear pyknosis in the hippocampus CA1 region compared to the WT group, but these pathological changes were significantly reduced by CDPS treatments (Figure 6F). These results demonstrated that CDPS treatments significantly reduced oxidative stress and brain pathology in the D-gal-induced aging model mice.

### CDPS treatment reduces peripheral inflammation and oxidative stress by maintaining gut microbial homeostasis in D-gal-induced model mice

Next, we analyzed if the changes in the composition of the gut microbiota were associated with increased peripheral inflammation and oxidative stress during aging. Towards this, we used a triple-antibiotic cocktail (ABX group) or cyclophosphamide (Cy group; also see Materials and methods) to ablate the gut microbiota or induce immunosuppression in the CDPS-treated aging model mice. The antibiotic treatment abrogated the beneficial effects of CDPS treatment in the aging model mice. We observed impaired learning and memory (Figure 7A), and alterations in the composition of gut microbiota (Figure 7B, 7C) in the ABX group mice compared to the CDPS-treated group. The above results indicate that even the administration of CDPS cannot increase the learning and memory ability of mice after changing the intestinal flora. Moreover, we observed increased levels of pro-inflammatory cytokines in the brain and the serum of ABX group mice compared to the CDPS group (Figure 7D–7N). The results of ABX group and CY group showed that after the intestinal flora and immune function were destroyed, even administration of CDPS could not improve the learning and memory ability of mice. These results suggested that CDPS treatment decreased peripheral inflammation, oxidative stress and cognitive decline in the D-gal-induced aging model mice by preventing gut dysbiosis.

**Figure 7:** **CDPS alleviates learning and memory by restoring homeostasis of the gut microbiota.** (**A**) Heat maps show long-term memory (preferential index*) and short-term memory (preferential index) in the WT, Mod, CM, ABX, and Cy groups of mice. (**B**) The relative abundance of top 10 gut microbial phyla in the WT, Mod, CDPS, ABX, and Cy groups of mice.(**C**) Venn diagram shows the number of bacterial operational taxonomic units (OTUs) in the WT, Mod, CDPS, ABX, and Cy groups of mice. (**D**–**I**) ELISA assays show levels of TNF-α, IL-2, IL-4, IL-10, SOD, and MDA in the serum of WT, Mod, CDPS, ABX, and Cy groups of mice. (**J**–**N**) Colorimetric assay results show the levels of AOPP, MDA, and LPO as well as activities of GSH-PX and SOD enzymes in the brains of WT, Mod, CDPS, ABX, and Cy groups of mice. Note: *p<0.05, **p<0.01, and ***p<0.001 compared to the WT group mice; #p<0.05, ##p<0.01, and ###p<0.001 compared to the Mod group mice. The data were analyzed by one-way ANOVA followed by the Dunnett's post hoc test. All values are represented as means ± SEM (n=15).

We then used the immunosuppressive drug, cyclophosphamide [24] to determine the role of inflammation in the beneficial effects of CDPS. Cyclophosphamide-treated CDPS mice (Cy group) showed impaired learning and memory ability, alterations in the gut microbiota composition, and aberrant levels of pro- and anti-inflammatory cytokines in the brain and serum compared to the wild-type and CDPS group mice. However, there is no significance comparing with model and ABX group. (Figure 7A–7N). These data demonstrate that alterations in the composition of the gut microbiota increase peripheral inflammation in the D-gal-induced aging model mice.

### CDPS prevents D-gal-induced aging by regulating amino acid metabolism

The immune system of the host is influenced by metabolites generated by the gut microbiota [25]. The fecal metabolites represent a functional readout of gut microbial metabolism and gut microbial composition [26]. Moreover, metabolites of the gut microbiota enter into blood circulation and impact host metabolism and health [26, 27]. A total of 1058 metabolites were identified in serum sample from fWT, Mod and CDPS mice. Then, we analyzed these metabolites using BioCyc, Kyoto Encyclopedia of Genes and Genomes (KEGG) and Human Metabolome Database (HMDB) and found that 65 metabolites were differentially expressed in the Mod group compared to the WT group. Furthermore, we found that the levels of 8 metabolites (creatinine, valine, L-(-)-Methionine, o-Toluidine, N-Ethylaniline, uric acid, proline and phenylalanine) significantly differed among the WT, Mod and CDPS groups. Pathway enrichment analysis of these 8 metabolites using MetaboAnalyst [28, 29] showed that these metabolites were related to arginine, histidine, arginine, proline, and purine metabolism (Figure 8A, 8B). 7 different metabolites of MOD group and CDPS group in WT group.

**Figure 8:** **CDPS inhibits peripheral inflammation and improves immune function by regulating amino acid and purine metabolism.** (**A**) Pathway enrichment analyses list of serum metabolites in the WT, Mod and CDPS group of mice. (**B**) Bubble chart of pathway enrichment analyses of serum metabolites in the WT, Mod and CDPS group of mice. (**C**) The serum concentration of various amino acids (creatinine, valine, L-(-)-Methionine, o-Toluidine, N-Ethylaniline, uric acid, and proline) in the ABX and Cy versus WT group of mice. (**D**, **E**) MetaboAnalyst results show the correlation between the differentially expressed metabolites and human diseases.

We then analyzed if changes in amino acid metabolism were related to alterations in the composition of the gut microbiota. We observed that 7 different metabolites of WT, Mod and CDPS groups (creatinine, valine, L-(-)-Methionine, o-Toluidine, N-Ethylaniline, uric acid, and proline) were significantly decreased in the ABX, Cy, and Mod groups compared to the WT and CDPS groups. Moreover, there is no significance between ABX and Cy group (Figure 8C). Finally, in order to explore there is a correlation between differential metabolism and other aging-related diseases. We analyzed the correlation between these seven differentially expressed metabolites and human diseases using the MetaboAnalyst database and found that these metabolites were associated with Alzheimer’s disease (*p*=0.00173; Figure 8D, 8E). Overall, these data suggested that CDPS protects against D-gal-induced aging by regulating amino acid metabolism.

## DISCUSSION

Progressive decline in cognitive function is a characteristic feature of aging. Previous studies showed that CDPS treatment significantly improved learning and memory in the aging model mice [30–33]. In this study, we demonstrated that CDPS treatment improved cognitive function by inhibiting peripheral inflammation and oxidative stress through restoration of gut microbial homeostasis in the D-gal-induced aging model mice (Figure 9). Sprague-Dawley rats fed with *Cistanche polysaccharides* showed increased growth of beneficial gut bacteria and enhanced gut microbial diversity [34]. CDA-0.05, a *Cistanche* neutral polysaccharide, improved the growth of probiotic *Lactobacilli* [22]. These data suggested that *Cistanche* polysaccharides improved homeostasis of gut bacteria.

**Figure 9:** CDPS alleviates cognitive decline by restoring homeostasis of the gut microbiota- brain axis in the D-gal induced aging model mice.

In this study, we demonstrated that CDPS has anti-inflammatory effects and improves cognitive ability of the aging model mice by modulating the abundance of gut bacterial genera such as *Bacteroidetes*, *Firmicutes,* and *Proteobacteria*. Hence, CDPS may be therapeutically beneficial for aging-related diseases by reshaping the composition of the gut microbiota [35, 36]. Moreover, previous studies have shown that the levels of inflammatory cytokines in the serum and colon are associated with the relative abundance of bacterial genera such as *Bacteroidetes*, *Firmicutes,* and *Proteobacteria* [37, 38]. Furthermore, gut microbial composition regulates brain function by modulating circulating levels of several cytokines [39–43]. Our results showed that CDPS treatment decreased the relative abundance of *Thermoplasmata, Bacilli*, unidentified *Actinobacteria*, *Fusobacteriia,* and unidentified *Elusimicrobia*, and increased the relative abundance of *Methanobacteria, Spirochaetia, Deltaproteobacteria,* unidentified*_Deferribacteres, Mollicutes, Nitrososphaeria, Anaerolineae, Erysipelotrichia,* and unidentified*_Cyanobacteria*.

Gut microbial metabolites are released into the blood stream and regulate the health and metabolism of the host [26, 27]_._ The gut microbial metabolites can be estimated by evaluating fecal metabolite composition, which changes with alterations in the composition of the gut microbes [44]. Recent studies have shown that plasma levels of citrulline, proline, arginine, asparagine, phenylalanine and threonine are associated with neurodegenerative disorders including Alzheimer’s disease [45, 46]. Our study showed that serum levels of creatinine, valine, L-methionine, o-Toluidine, N-ethylaniline, uric acid and proline were associated with D-gal-induced aging in mice.

The innate and adaptive arms of the immune system play a significant role in maintaining host-microbial homeostasis in the intestinal luminal surface [47]. The intestinal microbiota also play a significant role in regulating the central nervous system (CNS) and immunity by releasing cytokines and metabolites into the blood stream [48, 49]. The pro-inflammatory cytokines play a key role in several neurodegenerative diseases [50–52]. For example, age-related macular degeneration (AMD) and glaucoma is associated with extracellular accumulation of amyloid β (Aβ) and intracellular deposition of hyper-phosphorylated tau (p-tau) and iron in the retinal ganglion cells (RGC) [44]. Moreover, inflammation plays a significant role in pathogenesis associated with glaucoma [53]. Visual impairment is an early symptom of Alzheimer’s disease (AD) and is manifested before the onset of cognitive decline [54]. Our study demonstrated that CDPS protects against cognitive decline and peripheral inflammation by maintaining the homeostasis of the gut microbiota.

There are several limitations in this study. Firstly, the relationship between amino acid metabolism and composition of the gut microbiota is not well known. Secondly, the composition and molecular structure of CDPS is not known. Therefore, future studies are required to further explore the regulatory role of CDPS in alleviating AD through the gut microbiota-brain signaling axis.

In conclusion, our study demonstrated that CDPS improved cognitive ability in D-gal-induced aging model mice by restoring the homeostasis of gut microbiota, thereby restoring amino acid imbalance, peripheral inflammation, and oxidative stress. These findings suggest that CDPS is a potential therapeutic for patients with learning and memory disorders, especially those associated with gut dysbiosis.

## MATERIALS AND METHODS

### Preparation of CDPS

About 1.0 Kg of cleaned *Cistanche deserticola* was air-dried in the oven at 40° C and pulverized into crude powder. The powder was extracted in hot ethanol for 3 h. The residue was filtered through gauze to remove the filtrate and then diluted with water (8X) and refluxed sequentially for 2 h, 1.5 h, and 1 h at 90° C. At each time point, the solution was centrifuged to separate out the supernatant and combined with the brown-red filtrate. Then, the filtrate was concentrated under reduced pressure, cooled to room temperature, added slowly to 95% ethanol (3X), and allowed to stand at 4° C for 24 h. Then, the solution was centrifuged at 6000 r/min for 20 min at 4° C. The precipitate was collected after repeating water extraction and alcohol precipitation thrice. The precipitate was reconstituted in water, de-proteinized, dialyzed, and freeze-dried to get crude *Cistanche deserticola* polysaccharide (CDPS). The polysaccharide content was more than 90% as evaluated by ultraviolet spectrophotometry.

### Animal grouping and treatments

Eight-week old male Kunming mice (SCXK License No.2019-0010) were purchased from SPF Biotechnology Co. Ltd (Beijing, China), housed in a light and temperature-controlled room, and fed with food and water. All animal experiments were conducted according to protocols approved by the Institutional Animal Care and Use Committee of Inner Mongolia Medical University. The experiments were carried out according to the National Institutes of Health (NIH) Guide for the Care and Use of Laboratory Animals.

After 1 week adaptation to the new surroundings, 120 mice were divided into the following 7 groups: (1) wild-type control (WT); model group (150 mg/Kg/day D-gal; Mod); (3) CH: D-gal plus 100 mg/kg CDPS; (4) CM: D-gal plus 50 mg/kg CDPS; (5) CL: D-gal plus 25 mg/kg CDPS; (6) ABX group: antibiotics plus D-gal plus 50 mg/Kg CDPS; (7) Cy group: cyclophosphamide plus D-gal plus 50mg/kg CDPS.

The mice from the model, ABX, Cy, and CDPS groups received subcutaneous injections of saline-dissolved 150 mg/kg D-gal every day for 2 months. The WT group was subcutaneously injected with equal volume of saline for 2 months. The CDPS group mice were also administered daily with intragastric injections containing 100 mg/kg, 50 mg/Kg or 25 mg/Kg CDPS for 2 months. The ABX group mice received drinking water with 0.1 mg/mL ampicillin and 0.5 mg/mL streptomycin for 2 months in addition to D-gal and CDPS injections. Before administering D-gal, the mice received injections containing 0.1 mg/mL ampicillin, 0.5 mg/mL streptomycin, and 0.1 mg/mL colistin for 7 days in the ABX group. The Cy group mice received intraperitoneal injections of 20 mg/Kg cyclophosphamide every other day (q.o.d) for 2 months in addition to daily injections of D-gal and CDPS.

### Novel object recognition test

Conduct behavioral experiments after the last dose. The object recognition test involved familiarization, training, and testing stages. During familiarization stage, mice were habituated in an empty testing chamber for 10 minutes for two days. Then, on the third day (training day), two objects of the same size, shape, and color (A1 and A2) were placed on opposite ends of the chamber. Every mouse was then given 10 minutes to explore the two similar objects. After 1-hour (on the third day) and 24-hour (on the fourth day) training-to-testing intervals, one of the similar objects (A1 or A2) was replaced with a B or C object that is different in size, color and shape on the testing day. During testing stage, each mouse were tested for 5 minutes and the preferential index was calculated to determine the memory of novel object (B or C) recognition using the following formula: Preferential index=Time on object B or C/(Time on object B or C+Time on object A)×100%.

### Morris water maze test

Morris water maze test was performed in a round pool that was 45 cm in depth and 90 cm in diameter. The protocol described by Ruediger S, et al. (2011) [55] and Wood RA, et al. (2018) [56] was employed here. The water depth in the pool was 30 cm, and the temperature of water was 20±1° C. The platform was 6 cm in diameter and 1cm underwater. The time for training and testing was 60 s each. For training, we conducted four trials of 60 s each with a hidden platform every day for five continuous days. If the platform was not discovered by the mice in 60 s, they were guided to the platform, and placed on the platform for 5 s. During testing stage, the latency to reach the hidden platform in training and probe trial sessions, the number of crossing over the removed platform location, and the time spent in the target (platform) quadrant were recorded and analyzed.

### ELISA assays

The serum levels of pro-inflammatory cytokines such as IL-2(), IL-4, IL-10, and TNF-α were analyzed for each group of mice using ELISA kits purchased from Shanghai Yi Li Biological Technology Co., Ltd. (Shanghai, China) according to the manufacturer’ instructions. The activity of antioxidant enzyme, superoxide dismutase (SOD), and levels of lipid peroxidation product, malondialdehyde (MDA), in the serum of each group of mice was analyzed by assay kits purchased from the Nanjing Jiancheng Bioengineering Institute (Nanjing, China). The levels of advanced oxidation protein products (AOPP) in the murine hippocampus samples were estimated using ELISA kit from Shanghai Yi Li Biological Technology Co. Ltd. (Shanghai, China) according to the manufacturer’s instructions.

### Estimation of oxidative stress in murine brains

We homogenized 100 mg hippocampus tissue with 0.9 ml ice-chilled saline and the homogenate was centrifuged at 12000 rpm for 30 min at 4° C. The protein content in the supernatant was analyzed using the BCA Protein Assay Kit (Beyotime Biotechnology, Shanghai, China). The levels of lipid peroxidation (LPO) and malondialdehyde (MDA), and the activities of GSH-Px and SOD in the hippocampus samples were analyzed by colorimetry using kits from the Nanjing Jiancheng Bioengineering Institute (Nanjing, China) according to the manufacturer’s instructions.

### Gut microbiota composition

Fecal samples were collected from all mice and immediately stored at -80° C. The V3+V4 region of the 16S rRNA gene was sequenced using Illumina MiSeq (Beijing Novogene Co. Ltd., Beijing, China) and analyzed using the QIIME open platform to determine the gut microbiota profiles.

### LC/MS analysis of serum metabolites

Serum samples were incubated for 10 minutes with pre-chilled methanol in a ratio of 1: 3 to precipitate the proteins. The samples were centrifuged at 12000r/min for 15 minutes at 4° C. The supernatants were analyzed by Thermo Scientific Dionex UltiMate3000 Rapid Resolution Liquid Chromatography and QExactive mass spectrum. The chromatographic conditions are shown in Table 1. The analytes were separated in a XBridge BEH Amide chromatographic column (2.1×100 mm; Waters Co., Milford, MA, USA) using 0.1% formic acid and acetonitrile as mobile phases A and B, respectively. The flow rate was set at 0.4 ml/min, injection volume was 5 μl, and column temperature was set at 25° C (Table 1). The mass spectrum signals were obtained using the positive and negative ion scanning mode. The ion spray voltage and other specific MS parameters are shown in Table 2.

**Table 1:** Mobile phase elution gradient.

**Time (min)**	**Flow rate (mL/min)**	**A (%)**	**B (%)**
0	0.4	10	90
10	0.4	50	50
10.1	0.4	10	90

**Table 2:** Mass spectrometry source gas parameters and collision energy.

**M/Z**	**50-750**
IonSpray Voltage Floating (ESI+) (V)	4000
IonSpray Voltage Floating (ESI-) (V)	2200
Capillary Temperature (° C)	350
Sheath Gas (+) (arb)	40
Sheath Gas (-) (arb)	20
Max Spray Temperature (° C)	100
Probe Heater Temperature (+) (° C)	100
Probe Heater Temperature (-) (° C)	150

### Statistical analysis

Statistical analysis was performed using the SPSS 13.0 software (SPSS Inc., Chicago, Illinois, USA). The data plots were generated using GraphPad Prism 8.0.1 (GraphPad Software, La Jolla, California, USA). Partial least squares discriminant analysis (OPLS-DA) of SIMCA-P+13.0 (Umetrics, AB, Umeå, Sweden) and Principal Components Analysis (PCA) were used to assess normalized GC-MS spectral data. Variable Influence on Projection (VIP) values were used to identify significant variables with VIP values >1.0 and p< 0.05. These significant variables were used to identify the spectral peaks. Student's t-test was used to analyze differences between two groups of data. The taxonomic rank differential between groups was determined using Student’s test (v3.1.2; R programming language). The correlation between genera abundance and mouse behavior was calculated using Spearman correlation coefficients (R language). P < 0.05 was considered statistically significant. The data are presented as means±SEM.
